The article "The Effects of ERAS Concept Combined with Postoperative Leg Pad Elevation on Knee Enhancement, Quality of Life, and Pain in Sufferers after HTO Surgery" was retracted in 2023. Reasons: signs of a paper mill; suspected computer-generated content; unreliable results or conclusions; concerns about the data.

# The Effects of ERAS Concept Combined with Postoperative Leg Pad Elevation on Knee Enhancement, Quality of Life, and Pain in Sufferers after HTO Surgery

**DOI:** 10.1155/2022/8440977

**Published:** 2022-08-23

**Authors:** Wei Zhu, Qiong Li, Ju Huang

**Affiliations:** School of Nursing Wannan Medical College, Wuhu 241002, China

## Abstract

The effects of the enhanced recovery after surgery (ERAS) concept combined with postoperative leg pad elevation on knee enhancement, quality of life, and pain in sufferers after high tibial osteotomy (HTO) are investigated. A total of 98 sufferers who underwent high tibial osteotomy in our hospital from January 2020 to May 2021 were selected as the study subjects. Two sets of sufferers are randomly divided into the study set and the routine set by the random number table method, with 49 cases in each set. The contrast set is given routine nursing intervention, and the ERAS concept combined with self-made raising leg pad nursing is given to the study set on the basis of the contrast set. Efficacy, joint pain, knee function, SF-36 fraction, quality of life fraction, and psychological status fraction are observed in 2 sets. Experimental results show that for sufferers after HTO surgery, the application of the ERAS concept combined with leg pad nursing therapy can effectively enhance postoperative knee function and adverse mood, reduce postoperative pain, and enhance postoperative quality of life.

## 1. Introduction

Medial knee osteoarthritis can result from medial knee pain due to the medial alignment of the lower extremity. Medial compartment knee osteoarthritis is often treated with High tibial osteotomy (HTO). HTO can restore the biological axis of the knee joint to the correct position and effectively enhance the pressure on the medial tibial joint. Compression is beneficial to restore the damaged cartilage in the medial knee joint [1, 2]. The concept of enhanced recovery surgery is introduced by professor Henrik Kehlet of Denmark in 2001. The concept of enhanced recovery after surgery (ERAS) is based on the preparation of the sufferer's physical and mental conditions before surgery. It can reduce the physical and mental damage of sufferers during the whole process of surgery, enhance the postoperative recovery rate of sufferers, and enable sufferers to obtain the best prognosis, thereby effectively improving the recovery speed and satisfaction of sufferers [3, 4]. The use of the ERAS concept in most orthopedic operations has achieved good results. Some studies have found that ERAS in sufferers with orthopedic surgery can effectively reduce the postoperative complication rate, enhance the recovery time, and reduce adverse reactions of sufferers. The leg lift pad is a medical nursing pad, which is mainly used in the postoperative rehabilitation of fracture sufferers, but there are few clinical studies on the ERAS concept combined with the leg lift pad during early HTO surgery [5, 6]. This study analyzed the effect of the ERAS concept combined with postoperative leg raising on knee joint enhancement, quality of life, and pain in sufferers after HTO, in order to provide a theoretical basis for clinical rehabilitation of sufferers after HTO.

The article "The Effects of ERAS Concept Combined with Postoperative Leg Pad Elevation on Knee Enhancement, Quality of Life, and Pain in Sufferers after HTO Surgery" was retracted in 2023. Reasons: signs of a paper mill; suspected computer-generated content; unreliable results or conclusions; concerns about the data.

The rest of this paper is organized as follows: Section 2 discusses related work, followed by general information and statistical methods designed in Section 3.  Section 4 shows the experimental results, and Section 5 concludes the paper with summary and future research directions.

## 2. Related Work

At present, the main clinical therapy method for knee osteoarthritis is HTO surgery [7], which functions include biasing the sufferer's lower limb alignment, relieving joint pain, and ensuring the delay of knee replacement time, but in terms of the success rate of surgery, early postoperative functional exercise is extremely important. However, the pain, mentality, and resistance of sufferers all cause certain obstacles to postoperative joint function rehabilitation training [8].

Traditional rehabilitation programs are often based on general rehabilitation nursing models, without a unified scientific standard, resulting in poor efficacy and pertinence. At present, it has been confirmed by evidence-based medicine that fast recovery surgery plays an important role in clinical therapy as a theory for improving surgical measures [9]. Studies have shown that the concept of fast recovery surgery can effectively enhance the physical and mental health of sufferers and accelerate the recovery of sufferers' physical functions after surgery [10]. In this study, the concept of rapid rehabilitation was implemented for sufferers after HTO, and medical staff provided personalized pain care based on the distinct characteristics of sufferers. In addition, sufferers were given multimodal analgesia based on the combined effect of distinct means (improving the hospital environment, conducting psychological counseling, and health education). After therapy in distinct ways, there was a big disparity in the curative effect of the two sets of sufferers, mainly in that the curative effect of the study set was considerably higher than that of the contrast set; after 1 month of therapy, the VAS joint pain in both sets was enhanced, and the enhancement in the study set was significantly better. In the contrast set, the Lysholm fractions of the two sets of sufferers were enhanced, and the enhancement in the study set was significantly better than that in the contrast set (*P* < 0.05). The recovery of function thus relieves the sufferer's pain. The focus of ERAS was to assess the degree of postoperative pain in sufferers and take reasonable pain relief plans. Sufferers must learn related diseases and pain management knowledge under the guidance of medical staff, learn to correctly judge the degree of pain, and accurately express their feelings. At the same time, it can self-reduce postoperative pain through various nondrug measures (attention diversion and psychological suggestion) [11]. The self-made leg raising pad was used to support it, and the angle of the leg raising pad was set according to the actual situation of the sufferer, so as to ensure the freedom of movement of the sufferer, and at the same time prevented the sufferer's leg from shaking, reduced the occurrence of pain, and helped the sufferer recover [12].

The article "The Effects of ERAS Concept Combined with Postoperative Leg Pad Elevation on Knee Enhancement, Quality of Life, and Pain in Sufferers after HTO Surgery" was retracted in 2023. Reasons: signs of a paper mill; suspected computer-generated content; unreliable results or conclusions; concerns about the data.

Based on the sufferer's overall function, this study selected a combination of various methods for the sufferer's therapy plan, with the purpose of relieving the sufferer's postoperative pain, swelling, and psychological pressure. Because HTO can only relieve the knee joint pain caused by the force line, it has no effect on the pain caused by the internal damage of the knee joint and cannot adjust the arthritic area; the pain in the arthritic area, wound pain, and swelling of sufferers after HTO will all cause the appearance of the diseased limb [13]. At the same time, it should be noted that most of the selected examination subjects are the elderly, so during early rehabilitation therapy, attention should always be paid to the overall observation, focusing on the physical function of sufferers [14]. In this study, it was found that the SF-36 fractions of the two sets of sufferers were enhanced after therapy *P* < 0.05; after therapy, the Hamilton Anxiety (HAMA) scale and the Hamilton Depression (HAMD) scale fractions in the two sets were significantly decreased, and compared with the contrast set, the HAMA and HAMD fractions in the study set decreased significantly (*P* < 0.05). Because traditionally formulated rehabilitation nursing programs did not have scientific standards, the content of postoperative exercise lacks diversity, had no new ideas, and was poorly targeted. The formulation of the ERAS program should be based on scientific exercise therapy [15]. On the one hand, attention should be paid to speed up the recovery of tendons and bones in sufferers with anterior cruciate ligament rupture (ACLR) after surgery and to ensure normal internal fixation. The sufferer's use of the thigh pad to raise the thigh is conducive to determining the location of the lesion, the sufferer's limb was comfortable, and the venous return of the lower extremity was accelerated, thereby relieving the sufferer's limb swelling and pain and improving the happiness. When applied to sufferers after HTO, it can help sufferers with postural support and bone protrusion and other soft tissue protection, elevate the lower limb by 10–30 cm, and maintain the physiological bending of the lower limb. It was also suitable for lower-limb surgery, the tibia and fibula, and the femur [16].

The article "The Effects of ERAS Concept Combined with Postoperative Leg Pad Elevation on Knee Enhancement, Quality of Life, and Pain in Sufferers after HTO Surgery" was retracted in 2023. Reasons: signs of a paper mill; suspected computer-generated content; unreliable results or conclusions; concerns about the data.

It will promote blood circulation in the legs, leading to bedsore. In addition, the leg lift pad also has the following advantages: (1) the surface of the thigh pad has a groove design, which helps fix the position of the affected limb, accelerate the venous return of the lower limb, and relieve the swelling of the limb compared with other pads such as quilts and pillows. (2) The height of the thigh pad is adapted to the sufferer, which can accelerate blood circulation and reduce swelling and pain, and the material is comfortable, which greatly enhances sufferer satisfaction. (3) Thigh pads are affordable and more convenient and clean in nursing than other pads (quilts, pillows), which can reduce the life pressure of sufferers and the work of medical staff. (4) Thigh pads can not only avoid the trouble and pain caused by other pads to sufferers and medical staff but also can effectively enhance the quality of care. It is recommended to be widely used in clinical practice.

## 3. Examination Methods

### 3.1. General Information

A total of 98 sufferers who underwent high tibial osteotomy in our hospital from January 2020 to May 2021 were selected as the examination subjects. By using the random number table method, the two sets of sufferers are randomly divided into the study set and the routine set, with 49 cases in each set. In the examination set, there are 24 males and 25 females, with an age range of 31–58 years, an average age of (41.55 ± 4.71) years, and the ratio of left and right osteotomy directions is 23 : 26; the conventional set consisted of 28 males and 21 females. The age range is 30–59 years, the average age is (42.79 ± 3.58) years, and the ratio of left and right osteotomy directions is 25 : 24. The general clinical data such as age and gender are compared between the two sets, *P* > 0.05, and there is no extensive disparity between the two sets. All sufferers signed informed consent, and this study is approved by the medical ethics committee of our hospital. All sufferers included in the study signed the informed consent form. The therapy methods and detection methods used in this study are all known safe methods in the clinic; the general information and clinical data collected in this study are only used for examination decomposition, not for examination purposes. Other uses: If you have any discomfort during the treatment, please inform your doctor in charge in time to decide the next treatment plan. The whole treatment and observation period was 4 weeks. Please inform your doctor of the change of your condition. During the treatment, please do not use all other drugs and other treatment methods for this disease without authorization, and inform your doctor whether to use them.

The article "The Effects of ERAS Concept Combined with Postoperative Leg Pad Elevation on Knee Enhancement, Quality of Life, and Pain in Sufferers after HTO Surgery" was retracted in 2023. Reasons: signs of a paper mill; suspected computer-generated content; unreliable results or conclusions; concerns about the data.

### 3.2. Examination Methods and Observation Indicators

The contrast set is treated as follows: routine nursing interventions are given to this set of sufferers, including limb elevation, compression, drainage, close observation of skin color and temperature, peripheral circulation, and dorsal foot artery pulse.

The observation set is treated as follows: on the basis of the contrast set, the sufferers in this set are given the intervention of the *E* concept combined with the leg raised. The main contents are as follows: (1) First, reasonable psychological counseling should be given to sufferers before operation, and sufferers should be informed that there may be corresponding problems after operation. In case of severe reaction, an individualized rehabilitation plan should be implemented during hospitalization to reduce the sufferer's anxiety and fear of surgery. (2) After operation, the sufferer should be treated with a compression bandage first, and the sufferer's affected limb should be elevated. The self-made leg lift pad supports it. According to the actual situation of the sufferer, the angle of the leg lift pad is set to ensure that the sufferer's first thigh and second thigh can be supported and that the sufferer can move freely at all angles. At the same time, grooves are set at the support part of the sufferer's calf for parallel positioning to prevent the sufferer's calf from shaking left and right, causing the sufferer to suffer from pain (3) On the second day after the operation, the sufferer can be guided to perform muscle contraction training, including the abdominal muscles, gluteal muscles, and quadriceps. The exercise intensity is set to 10 per set, each for 10s; for the elderly, the overall body function should be taken care of as much as possible, and not only the lower limb muscles of the sufferer should be trained accordingly but also the sufferer should be instructed properly to perform upper limb and breathing training. We should help the sufferer perform shoulder circumference and muscle strength training through the action of the elastic band and also guide the sufferer to perform active flexion and extension exercises of the knee joint. The joints are flexed and extended as much as possible, but it should be noted that the sufferer should tolerate as much as possible, and then, the weight-bearing energy is increased in turn.

The article "The Effects of ERAS Concept Combined with Postoperative Leg Pad Elevation on Knee Enhancement, Quality of Life, and Pain in Sufferers after HTO Surgery" was retracted in 2023. Reasons: signs of a paper mill; suspected computer-generated content; unreliable results or conclusions; concerns about the data.

### 3.3. Observation Indicators

#### 3.3.1. Determination of Curative Effect

Criteria for clinical efficacy judgment are as follows [17]: ①Markedly effective: the sufferer's knee joint function is normal and completely recovered, the symptoms disappear completely, and daily activities are not restricted, and the X-ray examination shows that the Kellgren–Lawrence (KL) grading is 0. ②Effective: the sufferer's knee joint function tends to be normal, pain occasionally exists, symptoms basically disappear, and the degree of limitation of daily activities is low. X-ray examination shows that the KL classification is 2∼3. ③Ineffective: the sufferer has abnormal knee joint function, and pain often occurs. Symptoms do not enhance or even worsen, and daily activities are limited.

#### 3.3.2. Index Evaluation

There are five index evaluations that are as follows:

1. The pain of joints before and one month after therapy in the two sets is compared, and the Visual Analog Scale (VAS) [18] is used to evaluate them; the higher the fraction, the more severe the sufferer's knee pain.
2. The knee joint function of the two sets of sufferers before and after one month of therapy is compared [19]. The knee function fraction (Lysholm) is used to evaluate the knee joint function scale, and the scale fraction ranged from 0 to 10. The total score is 100 points, and the lower the fraction, the worse the knee joint function of the sufferer, and vice versa, the better.
3. To compare the disparity in SF-36 fractions between the two sets before and after therapy, the SF-36 scale [20] is evaluated from 8 aspects of social function, physiological function, physiological function, physical pain, overall health, vitality fraction, emotional function, and mental health. For evaluation, the total fraction score is 100 points, the higher the fraction is, the better the quality of life is.
4. The disparity in the fractions of the WHO quality of life scale (WHOQOL-BREF) [21] is compared between the two sets before and after therapy, society, and environment, with a total of 26 items, with a total fraction of 0 to 100. The higher the fraction, the higher the quality of life.
5. The psychological state fractions of the two sets before and after therapy are compared [22, 23], and the degree of anxiety and depression of sufferers are evaluated by the HAMA scale and the HAMD scale. The HAMD fraction has 24 subitems, each with a fraction of 0 to 4, and the higher the fraction, the more severe the depression; the HAMA fraction has 14 subitems, each with a fraction of 0 to 4, and the higher the fraction, the more severe the anxiety.

The article "The Effects of ERAS Concept Combined with Postoperative Leg Pad Elevation on Knee Enhancement, Quality of Life, and Pain in Sufferers after HTO Surgery" was retracted in 2023. Reasons: signs of a paper mill; suspected computer-generated content; unreliable results or conclusions; concerns about the data.

### 3.4. Statistical Methods

In this study, a corresponding database is established for all data, and all the data processing databases were entered into SPSS 26.0. The normal test of the measurement data line is expressed as ($\bar{x}\pm s$) [24–27]. The data that conform to the normal test are between groups *F*. Multiple repeated measurements are decomposed by *MANOVA* spherical decomposition [28], and the data between groups are tested by the independent samples *t* test. The paired sample *T* test is used for intraset data, and the Mann–Whitney *U* test is used for non-normal data. The rate is expressed as %, and the test is *χ2*. When *P* < 0.05, the disparity between data is considered statistically significant.

## 4. Experimental Results

### 4.1. Clinical Efficacy Comparison between the Two Sets

Table 1 is the comparison of clinical efficacy between the two sets. As shown in Table 1, there is an extensive disparity in the efficacy of the two sets, mainly manifested as the efficacy of the study set is significantly higher than that of the contrast set (*P* < 0.05) after distinct therapy methods.

### 4.2. Comparison of Sufferers' Joint Pain before Therapy and One Month after Therapy

Table 2 is the comparison of joint pain before therapy and one month after therapy. In Table 2, “a” represents comparison before therapy, *P* < 0.05. It can be seen from Table 2 that the VAS joint pain is higher in 2 sets, and the disparity is not statistically significant (*P* > 0.05) before therapy. The VAS joint pain is enhanced in both sets, and the enhancement in the study set is significantly better than that in the contrast set (*P* < 0.05) after therapy.

### 4.3. Comparison of the Knee Function of Sufferers before and after Therapy

Table 3 is the comparison of the knee function before and after therapy ($\bar{x}\pm s$). In Table 3, “a” represents comparison before therapy, *P* < 0.05.  Figure 1 is the comparison of the knee function before and after therapy. It is clearly evident from Table 3 and Figure 1 that the Lysholm fraction of the knee function in 2 sets is lower, and the disparity is not statistically significant (*P* > 0.05) before therapy. The Lysholm fraction of the knee function is enhanced in both sets, and the enhancement in the study set is significantly better than that in the contrast set (*P* < 0.05) after therapy.

### 4.4. Comparison of the SF-36 Fraction between 2 Sets before and after Therapy

Table 4 is the comparison of the SF-36 fraction between the two sets before and after therapy.  Figure 2 is the comparison of the SF-36 fraction between the two sets before and after therapy. Through the above experimental results, it can be observed that there is no significant difference in the SF-36 fraction between the two sets (*P* > 0.05) before therapy. The SF-36 fractions in both sets are enhanced, and the enhancement in the study set is significantly higher than that in the contrast set (*P* < 0.05) after therapy.

The article "The Effects of ERAS Concept Combined with Postoperative Leg Pad Elevation on Knee Enhancement, Quality of Life, and Pain in Sufferers after HTO Surgery" was retracted in 2023. Reasons: signs of a paper mill; suspected computer-generated content; unreliable results or conclusions; concerns about the data.

### 4.5. The Comparison of the WHOQOL-BREF Fraction between the Two Sets before and after Therapy

Table 5 is the comparison of the WHOQOL-BREF fraction between the two sets before and after therapy. In Table 5, “a” represents comparison before therapy, *P* < 0.05. It can be seen from Table 5 that the WHOQOL-BREF fractions and the total fractions of psychology, physiology, society, and environment in 2 sets show no significant difference (*P* > 0.05) before therapy. The WHOQOL-BREF fractions and total fractions of the two sets are significantly enhanced, and the enhancement in the study set is significantly higher than that in the contrast set (*P* < 0.05) after therapy.

### 4.6. The Comparison of Psychological Status Fractions between the Two Sets before and after Therapy

Table 6 is the comparison of psychological state fractions between the two sets (fraction, $\bar{x}\pm s$). In Table 6, “a” represents comparison before therapy, *P* < 0.05.  Figure 3 is the comparison of psychological state fractions between the two sets before and after therapy. Through the above experimental results, it can be observed that the HAMA and HAMD fractions are not significantly different between the two sets before therapy (*P* > 0.05). The HAMA and HAMD fractions in the two sets decreased significantly after therapy, and the HAMA and HAMD fractions in the study set decreased significantly compared with the contrast set (*P* < 0.05).

## 5. Conclusion and Future Work

Although this study has achieved certain examination results, it still has certain limitations because only 98 sufferers are included in this study, and there are only 49 sufferers in each set after setting. Too few cases may lead to certain bias in the results. Therefore, in future examination, the sample size should be further expanded to analyze the efficacy and value of the ERAS concept combined with leg raising in sufferers after HTO. For sufferers after HTO, the application of the ERAS concept combined with leg raising nursing therapy can effectively enhance postoperative knee function and negative emotions, reduce postoperative pain, and improve patients' quality of life. The research is worthy of clinical application.

The article "The Effects of ERAS Concept Combined with Postoperative Leg Pad Elevation on Knee Enhancement, Quality of Life, and Pain in Sufferers after HTO Surgery" was retracted in 2023. Reasons: signs of a paper mill; suspected computer-generated content; unreliable results or conclusions; concerns about the data.

## Figures and Tables

**Figure 1:** Comparison of the knee function before and after therapy.

**Figure 2:** Comparison of the SF-36 fraction between the two sets before and after therapy.

**Figure 3:** Comparison of psychological state fractions between the two sets before and after therapy.

**Table 1:** Comparison of clinical efficacy between the two sets (*n* (%)).

Set	Effective	Efficient	Invalid	Total efficiency
Study set (*n* = 49)	25	22	2	47（95.92）
Contrast set (*n* = 49)	16	14	19	30(61.22)
*χ2*				17.526
*P*				＜0.001

**Table 2:** Comparison of the joint pain before therapy and one month after therapy ($\bar{x}\pm s$).

Set	Before therapy	After therapy
Study set (*n* = 49)	6.92 ± 1.12	1.26 ± 0.45^a^
Contrast set (*n* = 49)	6.97 ± 1.15	2.33 ± 0.56^a^
*T*	0.471	−11.633
*P*	0.709	＜0.001

**Table 3:** Comparison of the knee function before and after therapy ($\bar{x}\pm s$).

Set	Lysholm	
	Before therapy	After therapy
Study set (*n* = 49)	55.62 ± 8.57	87.56 ± 11.57^a^
Contrast set (*n* = 49)	56.12 ± 8.58	72.78 ± 9.82^a^
*t*	−0.8123	8.526
*P*	0.410	＜0.001

**Table 4:** Comparison of the SF-36 fraction between the two sets before and after therapy (fraction, $\bar{x}\pm s$).

Set	SF-36		*t*	*P*
	Before therapy	After therapy		
Contrast set (*n* = 49)	50.21 ± 4.57	71.32 ± 5.48	18.943	< 0.001
Study set (*n* = 49)	49.78 ± 5.14	83.12 ± 5.11	−29.454	< 0.001
*t*	0.402	−10.149		
*P*	0.688	< 0.001		

**Table 5:** Comparison of the WHOQOL-BREF fraction between the two sets before and after therapy (fraction, $\bar{x}\pm s$).

Project	Before therapy		*t*	*P*	After therapy		*t*	*P*
	Contrast set (*n* = 49)	Study set (*n* = 49)			Contrast set (*n* = 49)	Study set (*n* = 49)		
Psychological	10.45 ± 3.43	10.38 ± 3.54	0.091	0.927	12.47 ± 2.12^a^	16.56 ± 1.87^a^	−9.327	＜0.001
Physiological	15.36 ± 3.52	15.28 ± 3.48	0.104	0.917	16.15 ± 3.12^a^	18.43 ± 3.73^a^	−3.017	0.003
Social	12.61 ± 4.76	12.57 ± 4.68	0.039	0.969	13.26 ± 3.45^a^	15.77 ± 3.64^a^	−3.223	0.002
Environment	15.36 ± 4.32	15.26 ± 4.43	0.104	0.917	16.57 ± 2.34^a^	18.69 ± 2.07^a^	−4.374	＜0.001
Total fraction	53.77 ± 10.36	54.38 ± 10.42	−0.267	0.790	58.74 ± 11.67^a^	71.23 ± 12.32^a^	−4.740	＜0.001

**Table 6:** Comparison of psychological state fractions between the two sets (fraction, $\bar{x}\pm s$).

Set	HAMA		HAMD	
	Before therapy	After therapy	Before therapy	After therapy
Contrast set (*n* = 49)	23.78 ± 2.44	17.32 ± 2.33^a^	35.24 ± 1.89	26.32 ± 2.43^a^
Study set (*n* = 49)	24.01 ± 2.53	9.07 ± 2.21^a^	35.33 ± 2.01	18.45 ± 2.32^a^
*t*	−0.421	16.554	−0.210	15.094
*P*	0.675	＜0.001	0.834	＜0.001

## Data Availability

The simulation experiment data used to support the findings of this study are available from the corresponding author upon request.
